This article has been retracted.

# The Current Situation and Influencing Factors of the Alarm Fatigue of Nurses' Medical Equipment in the Intensive Care Unit Based on Intelligent Medical Care

**DOI:** 10.1155/2021/9994303

**Published:** 2021-07-03

**Authors:** Yunxia Zhao, Minlin Wan, Huisong Liu, Mei Ma

**Affiliations:** ^1^Intensive Care Unit, Qingdao Municipal Hospital, Qingdao 266011, Shandong, China; ^2^Nursing Department, Qingdao Municipal Hospital, Qingdao 266011, Shandong, China

## Abstract

After rapid development and reform, the health level and medical diagnosis and treatment capabilities of Chinese residents have been significantly improved, and high-quality medical resources have significantly improved the life safety and health of the masses. As the most concentrated area of medical equipment in the hospital, the intensive care unit produces the most alarms during the operation of the equipment. The intensive care unit nurses are responsible for heavier nursing work, and the problem of alarming in other departments is more prominent. Therefore, this paper presents an analysis and research on the current situation and influencing factors of the alarm fatigue of nurse medical equipment in the intensive care unit based on intelligent medicine. This article uses a variety of related methods such as literature data method and questionnaire survey method to deeply study the theoretical knowledge of intelligent medical treatment, medical equipment alarm fatigue device, and so on. The logistic regression analysis method is introduced to classify its influencing factors, and the analysis experiment on the influencing factors of the medical equipment alarm fatigue of nurses in the intensive care unit is designed. The nurses' cognition of clinical alarms and the analysis of clinical alarm fatigue questionnaire data are studied. The alarm fatigue of nurses in the intensive care unit is at a severe level, which needs to be taken seriously in the intensive care unit. Unmarried, high-level positions, long working years, high professional titles, and high education are negatively correlated with alarm fatigue (*P* < 0.05), and those without an alarm habit are positively correlated with alarm fatigue (*P* < 0.05), and the number of night shifts per month is related to alarm fatigue. There is no correlation between them (*P* > 0.05).

## 1. Introduction

In recent years, the emergence and development of smart medical care has played an important role in improving doctors' diagnosis and treatment capabilities and narrowing the gap between urban and rural medical services. However, the penetration rate of smart medicine in medical institutions at all levels in our country is still not ideal. It has not yet formed a strong support for promoting the balanced distribution of high-quality medical resources and promoting the improvement of the diagnosis and treatment level of primary medical institutions. Therefore, this article focuses on the research of related influencing factors based on intelligent medical treatment and analyzes the main influencing factors in combination with key factors that affect the diagnostic accuracy and comprehensibility of the medical equipment alarm fatigue of nurses in the intensive care unit.

Alarm fatigue is a complex and uncontrollable cognitive process. It is the result of changes in human cognition and attention to adapt to the surrounding environment. Alarm fatigue cannot be simply regarded as an overcontact alarm. As the most concentrated area of medical equipment in the hospital, the intensive care unit produces the most alarms during the operation of the equipment. The intensive care unit nurses are responsible for heavier nursing work, and the problem of alarming in other departments is more prominent.

Li F alert fatigue is a key safety issue because it increases workload and weakens the operator's situational awareness. A design method to enhance the interaction between the alarm system and the operator is proposed. Taking the input of VTS personnel as the basic design requirements, a user-demand-driven design framework is proposed. It integrates quality function deployment, creative problem solving theory, and software quality characteristics into three design stages. In the first stage, user requirements are obtained through analysis of the current workflow. The second stage studies the specific nonfunctional design requirements and contradictions of the ship alarm system. In the third stage, the innovative principle of the contradiction matrix is analyzed. Through a case study, the framework was verified and explained, and a conceptual design of an intelligent ship alarm system was proposed. However, the intelligent ship alarm system he designed is not suitable for use in intensive care units [1]. Early active mobilization and rehabilitation in the Tipping C J Intensive Care Unit (ICU) are being used to prevent the long-term functional consequences of critical illness. Some experts aim to determine the impact of active mobilization and rehabilitation in the ICU on mortality, function, mobility, muscle strength, quality of life, survival days and discharge to 180 days, ICU and hospital stay, duration of mechanical ventilation, and discharge destination. The results are linked to the World Health Organization's international functional classification framework. Methods: the PRISMA checklist guides the systematic review and meta-analysis of randomized controlled clinical trials. Results: 14 studies of different quality including 1753 patients were reviewed. Active mobilization and rehabilitation had no effect on short-term or long-term mortality (*P* > 0.05). The analysis showed that active mobilization and rehabilitation resulted in greater muscle strength (body function) using the medical research committee's total score (average difference 8.62 points) when discharged from the intensive care unit. Related scholars' research showed the condition of the ICU intensive care unit. However, there is no more research on the alarm processing in the intensive care unit [2]. Since Kim has spread rapidly as a new communication mode, people have conducted a lot of research on various applications of the Internet of Things. In particular, people have done a lot of research on various applications of the Internet of Things. Yes, people's interest in smart medical systems is increasing day by day. In smart medical systems, a large number of medical devices are distributed in popular areas such as stations and medical centers. This high-density distribution of medical devices will cause serious degradation of communication performance, which is called coexistence. Problem: when the smart medical system has a coexistence problem, it may not be able to guarantee the reliable transmission of patient biological information, endangering the patient's life safety. Therefore, the coexistence problem in the smart medical system must be solved. Some people proposed a smart medical system based on the Internet of Things distributed coexistence mitigation scheme, which can dynamically avoid interference in the case of coexistence and ensure reliable communication. In order to evaluate the performance of the proposed scheme, they conducted a lot of simulations through comparison with IEEE802.15.4. However, the experimental results are not carried out under the control of variables, so there are still some problems in practical applications [3].

This article mainly studies the current situation and influencing factors of the alarm fatigue of nurse medical equipment in the intensive care unit based on intelligent medical care. First, it deeply learns theories and logistic regression analysis methods of intelligent medical care, intensive care unit, and alarm monitoring equipment and then designs questionnaire survey, experimental research on multiple nurses in Y hospital, and finally analyzes the nurses' awareness of medical equipment alarms and the influencing factors of alarm fatigue. The innovation of this article is that the previous research focuses on the research of instruments and equipment, but the research direction of this article focuses more on the research of nurses' influence factors on alarm fatigue, so that there is a better direction to improve the quality of nurses' service and protect patients' safety of life.

## 2. Research Methods Based on the Current Situation and Influencing Factors of the Alarm Fatigue of Nurse Medical Equipment in the Intensive Care Unit Based on Intelligent Medical Care

### 2.1. Smart Medical

Intelligent medical treatment refers to an intelligent system developed based on artificial intelligence technologies such as machine learning and deep learning to support doctors' diagnosis and treatment [4]. The main purpose is to improve the work efficiency and clinical ability of doctors. Its core is to process medical data and extract medical knowledge through artificial intelligence technology.

With the rapid development of information technologies such as big data and deep learning, medical knowledge mining, disease risk prediction, and disease-assisted diagnosis based on natural language, machine learning, and deep learning technologies have become the key research objects of artificial intelligence research [5]. The decision-making method of intelligent medical assistance diagnosis is one of the research hotspots. The use of medical information technology has become an important way to improve the level of medical service and medical quality [6]. In order to discover the key factors that influence the adoption behavior of medical information technology and its related applications by adopters, so as to promote the use and promotion of medical information technology, a large number of researchers have conducted research on the influencing factors of medical information technology adoption behavior based on theories such as technology adoption behavior [7, 8]. The medical information technology adopted in the research mainly includes medical information systems and services such as clinical information systems, mobile medical treatment, electronic medical records, and electronic health records [9]. According to the different subjects (users) of survey adoption, medical information technology adoption research can be divided into three categories: medical institutions, patients (consumers), and medical staff. Among them, patients (consumers) and medical staff are the main research objects of researchers.

### 2.2. Intensive Care Unit and Alarm Monitoring Equipment

The intensive care unit is the unit for intensive treatment of critically ill patients in various hospitals, and it is the department with the most intensive equipment. Medical equipment such as monitors, ventilators, and micro-pumps keep beeping to attract the attention of medical staff. Before 1983, there were no more than 6 types of clinical alarms used to monitor patients, but by 2011 this number had increased to more than 40 types [10]. Although there are thousands of alarm messages every day in the hospital, 85%–99% of them are alarms that do not need to be processed or are erroneous [11]. Therefore, in 2014, ECRI accused the life-saving equipment technology as a “problem,” which shows that frequent alarms have caused trouble to clinical work [12]. In 2015, ECRI listed the alarm hazard as the first of the “Ten Health Technology Hazards” first formulated since 2007 [13].

A series of problems caused by the alarm have attracted more and more attention from various countries. At the same time, frequent alarms will cause healthcare personnel not to intervene or delay processing the alarm prompts, and sometimes they may completely ignore or reset the alarm information. This phenomenon is called “alarm fatigue” [14, 15]. Alarm fatigue may cause adverse events and serious threats to the lives of patients and eliminate the waste of nursing resources caused by a large number of false alarms [16]. Therefore, it is particularly important to analyze the influencing factors of nurses' clinical alarm cognition in the intensive care unit, which can provide a basis for effectively reducing nurses' alarm fatigue, guiding alarm management, and quality planning. As an important part of patient vital signs monitoring, monitors have been widely used in various clinical departments, and monitors have the highest proportion of false alarms. Now, we will summarize the literature on monitor alarms that we have searched for and make a summary as follows.

#### 2.2.1. Alarm Classification

At present, there is no universally recognized standard for the classification of medical equipment alarms. According to the validity, the alarms are classified into true positive alarms, true negative alarms, false negative alarms, and false positive alarms [17, 18]. True positive alarm is to indicate that the patient is truly abnormal, which is a true alarm that is meaningful for the treatment of the patient; true negative alarm refers to the situation where the patient has an abnormal condition without any alarm [19]; false positive alarms refer to useful alarms that are not related to the condition of clinical patients, including alarms for technical problems of the instrument; false negative alarms refer to false alarms that cannot reflect changes in the patient's status. According to the actual situation of the device, from the point of view of whether the alarms that occur are interfering, they can be divided into action and nonaction [20]. This is directly related to the patient's life insurance and is an alarm that must be handled by medical personnel and is also called an effective alarm. Alarms that do not work must include alarms generated by moving objects and technical alarms [21]. Although scholars have made different definitions of clinical alarms, in the end they all regard alarms that can truly reflect the fluctuations in the vital signs caused by the changes in the patient's condition as correct alarms. On the contrary, alarms that are not related to medical facilities and patients become false alarms or alarms.

#### 2.2.2. The Impact of the Alarm

There are many types of alarms in the intensive care unit. Studies have shown that 32 devices in the intensive care unit can generate 45 different types of alarms. According to previous studies, it is found that nurses can only distinguish between 6 and 14 different types of alarms. These alarms have brought great trouble to the nurses' work [22, 23]. At present, there is no unified international standard for medical equipment alarms. When equipment manufacturers are pursuing instrument sensitivity, they often ignore the specificity of alarms, resulting in a large number of false alarms [24]. At the same time, in order to prevent accidents caused by ignoring the alarm, the manufacturer sets the default alarm setting for the instrument. When the default setting does not match the patient's condition, it will also cause a large number of false alarms and meaningless alarms.

#### 2.2.3. Alarm Fatigue

Alarm fatigue is usually related to medical institutions that issue multiple alarms due to various reasons such as effective alarm information and invalid false alarm information that reduce the nurse's ability to respond and the effectiveness of treatment [25]. If the machine cannot provide effective alarm information, it will make the medical staff visually fatigued and increase the risk of the patient during the treatment [26, 27]. Under normal circumstances, nurses are the first responders to clinical medical equipment alarms. The degree of importance and response speed of nurses to medical equipment alarms directly affects the safety of patients during hospitalization. Nurses, as the direct managers of clinical alarms, have not been in the current research. At present, the research and management of domestic alarm response fatigue is relatively slow, and the research mainly focuses on information equipment and technology. There are almost no reports on the knowledge of medical experts, the analysis of human factors, and the countermeasures against alarm and fatigue [28].

Figure 1 is a picture of the intensive care unit of a hospital.

### 2.3. Logistic Regression Analysis Method

The logistic regression algorithm is a classic binary classification algorithm. It belongs to a generalized linear model. It is often used in data mining, disease diagnosis, economic forecasting, and other directions. The difference from multiple linear regression models is the type of dependent variable. Logistic regression is used when the binomial distribution is followed, and multiple linear regression model or logistic regression is selected when the dependent variable is a continuous variable. Logistic regression is a classic algorithm that is easy to understand and implement. It can be used for classification as well as for predicting probability. In data mining, logistic regression is generally preferred, and then other algorithms are considered. Because the model is simple, logistic regression has a strong “resilience” when faced with fast-updated data. When the analysis target is a binary classification problem, the logistic regression algorithm is usually preferred.

The derivation of the logistic regression formula is relatively simple. Before introducing logistic regression in detail, first introduce the Sigmoid function. The formula is as follows:

(1) $$\begin{array}{c} T\left(x\right)=\frac{1}{\left(1+e^{-x}\right)},\;x\in R. \end{array}$$

From formula (1), we can see that the value of the independent variable *z* is any real number, and the value range is [1,0]. Therefore, the function of this function is consistent with any input [1, 0] in the space, and the projection value obtained by linear regression corresponds to the input function. After adjusting the probability threshold, the probability value is converted into two classification tasks. Calculate regression based on linear regression and apply this function. Such input is used to convert digital output into probability. This shows that it is not a regression problem, but a classification problem.

Let the prediction function be

(2) $$\begin{array}{c} p_{\mu }\left(x\right)=h\left(\mu^{T}x\right)=\frac{1}{\left(1+e^{-\mu^{T}x}\right)}, \end{array}$$

where *μ* is the estimated parameter.

(3) $$\begin{array}{c} \mu_{0}+\mu_{1}x_{1}+\mu_{2}x_{2}+\cdots +\mu_{n}x_{n}=\sum_{i=1}^{n}\varsigma_{1}x_{1}. \end{array}$$

Then, the classification task can be expressed as

(4) $$\begin{array}{c} \left\{\begin{array}{c} Q\left(y=1|x;\varsigma \right)=p_{\varsigma }\left(x\right),\\ Q\left(y=0|x;\varsigma \right)=1-p_{\varsigma }\left(x\right). \end{array}\right. \end{array}$$

After integrating equation (4), we get

(5) $$\begin{array}{c} Q\left(y|x;\varsigma \right)=p_{\varsigma }\left(x\right)\cdot {\left[1-p_{\varsigma }\left(x\right)\right]}^{1-y}. \end{array}$$

For the binary classification task (0,1), when the category is 1, that is, when *y* = 1, the above formula is *Q*=*p*_*ς*_(*x*), and when the category is 0, that is, when *y* = 0, the above formula is *Q*=1 − *p*_*ς*_(*x*).

#### 2.3.1. Influencing Factor Selection Method Based on Information Entropy

Information is a broad and systematic concept. In order to measure information, some scholars have proposed information entropy. Information entropy is a concept that measures the amount of information from the perspective of statistics and probability, and it has certain advantages especially for the measurement of discrete information. From the point of view of sample selection, only the sample with the greatest stability or the least uncertainty can express as much information as possible. In this section, the size of information entropy is used as a measure to determine whether the sample set contains the maximum amount of information.

According to the research needs of this article, a sample set with a large amount of sample information is selected according to the requirements to solve the data balance problem. Suppose a random variable *X*; *t*(*x*) represents the probability value of the random variable *X* at *x*; then the information entropy can be expressed by the following equation:

(6) $$\begin{array}{c} W\left(x\right)=-\sum t\left(x\right)\cdot \;\log\;t\left(x\right),\;i=1,2,3,\ldots ,n. \end{array}$$

If the random variable *X* is a continuous value, then equation (6) can be written as

(7) $$\begin{array}{c} W\left(x\right)=-\int_{x}^{\infty }t\left(x\right)\cdot \;\log\;t\left(x\right)\text{d}x. \end{array}$$

The problem of variable probability estimation is a basic problem in statistics. Kernel density estimation (also known as Parzen window estimation) is commonly used to solve this problem. Studies have shown that the method of using the kernel density estimation method to obtain the probability distribution of the sample and then obtaining the Shannon entropy (Shannon) according to the probability distribution is very cumbersome, especially in the multi-dimensional personal credit score evaluation selected in this article, the solution process is more complicated, and similarly the Renyi entropy instead of information entropy will greatly reduce the computational complexity. In information theory, the Renyi series includes Shannon entropy, Hartley entropy, minimum entropy, and conflict entropy. Renyi entropy is an extension of Shannon entropy, and it is also q-order generalized entropy. Renyi entropy (Renyi) is defined as follows:

(8) $$\begin{array}{c} W_{R}\left(U\right)=\frac{1}{1-b}\log\sum_{x}t_{i}{\left(x\right)}^{b},\;b>0,b\neq 1. \end{array}$$

In the formula, *U* is a discrete variable, *b* represents the order of Raney entropy, and *t*_*i*_(*x*) represents the probability of variable *x*. At that time *b*⟶1, WR was Shannon entropy. When *b* = 2, it is the quadratic Raney entropy. Correspondingly, the quadratic Raney entropy of continuous variables is as follows:

(9) $$\begin{array}{c} W_{R}\left(x\right)=-\log\int t_{i}{\left(x\right)}^{2}\text{d}x. \end{array}$$

With a sample set *U*=*x*_1_, *x*_2_,…, *x*_*n*_, let us use *R*(*r*)=∑_*x*_*r*(*x*)^2^ the kernel density to estimate:

(10) $$\begin{array}{c} \hat{R}\left(x\right)=-\frac{1}{n}\sum_{x_{i}\in U}l_{\beta }\left(x,x_{i}\right). \end{array}$$

Among them, *i*=1,2,…, *n*, *l*_*β*_(*x*, *x*_*i*_) represents *β* the kernel density function whose bandwidth *x*_*i*_ is the center of function. Generally, if the sample mean is used as an estimate, then there is

(11) $$\begin{array}{c} \hat{r}\left(r\right)=\frac{1}{n}\sum_{x_{i}\in U}\hat{r}\left(x\right)=\frac{1}{n^{2}}L^{T}KL. \end{array}$$

Therefore,

(12) $$\begin{array}{c} Y_{R}\left(x\right)=-\log\int r_{i}{\left(x\right)}^{2}\text{d}x=-\log\left(\frac{1}{n^{2}}L^{T}KL\right). \end{array}$$

In the formula, *K* represents the kernel density matrix of *n* ∗ *n*, and *L* represents the vector of *n* ∗ 1, from which the Raney entropy of the sample can be calculated.

#### 2.3.2. Principal Component Analysis Method

Principal component analysis is one of the most frequently used dimensionality reduction methods. The basic idea is to finally convert a series of related indicators into indicators without new relationships through rotation. The new indicator is a linear combination of the old indicator. The greater the variance after combination, the more information it represents.

Use principal components to extract sample information: suppose there are *n* samples in the original data set *X*, and each sample has *p* indicators. The idea of principal component analysis is to effectively combine these *p* indicators into new *m* indicators in a certain way (*m* < *p*), that is, the linear combination of *m* indicators represents the original *p* indicators, and the process is as follows:

(13) $$\begin{array}{c} T=\left[\begin{array}{ccc} T_{11} & \cdots & T_{1p}\\ \vdots & \ddots & \vdots \\ T_{n1} & \cdots & T_{np} \end{array}\right]=\left[\begin{array}{ccc} T_{1} & \cdots & T_{p} \end{array}\right], \end{array}$$

among them,

(14) $$\begin{array}{c} T_{j}=\left[\begin{array}{c} T_{1j}\\ T_{2j}\\ \vdots \\ T_{nj} \end{array}\right],\;j=1,2,\ldots ,p. \end{array}$$

Relinearly combine these *p* variables into *m* variables:

(15) $$\begin{array}{c} \left\{\begin{array}{c} D_{1}=\alpha_{11}T_{1}+\alpha_{12}T_{2}+\cdots +\alpha_{1P}T_{P}\\ D_{2}=\alpha_{21}T_{1}+\alpha_{22}T_{2}+\cdots \alpha_{2P}T_{P}\\ \;\;\;\;\;\;\cdots \\ D_{m}=\alpha_{m1}T_{1}+\alpha_{m2}T_{2}+\cdots \alpha_{mp}T_{p}. \end{array}\right. \end{array}$$

In the formula, *D*_*m*_ is the *m*-th new index obtained after principal component transformation. Principal component analysis extracts indicators according to indicator contribution rate and cumulative contribution rate: (1) contribution rate: the ratio of the eigenvalue of the *i*-th principal component to the sum of all eigenvalues in the covariance matrix. The larger the ratio of *i*, the greater the amount of original data information represented by the *i*-th index. The eigenvalue of the i-th principal component is *iλ*; then the contribution rate is expressed as

(16) $$\begin{array}{c} \beta_{i}=\frac{\nu_{i}}{\sum_{i=1}^{p}\nu_{i}}. \end{array}$$

Cumulative contribution rate: the ratio of the sum of eigenvalues of the first *k* principal components to the sum of all eigenvalues. The larger the value of the cumulative contribution rate, the more information it contains. The cumulative contribution rate is usually used to measure the number of final selected indicators. Generally speaking, at least the number of indicators with a cumulative contribution rate of 80% or more is of greater research significance.

(17) $$\begin{array}{c} C_{K}=\frac{\sum_{i=1}^{k}\nu_{i}}{\sum_{i=1}^{p}\nu_{i}}. \end{array}$$

## 3. Based on the Research Experiment of the Current Situation and Influencing Factors of the Alarm Fatigue of Nurse Medical Equipment in the Intensive Care Unit

### 3.1. The Experimental Research Object on the Influence of the Alarm Fatigue of the Nurse Medical Equipment in the Intensive Care Unit

The research subjects used the convenience sampling method. From September 1, 2019, to September 10, 2019, among the 254 nurses in the intensive care unit registered in the four tertiary hospitals in Y city, 220 people who met the inclusion criteria were issued questionnaires. 220 questionnaires were distributed, 215 points were returned, and the recovery rate was 98%.

(i) Inclusion criteria
  1. Registered nurse in intensive care unit
  2. Working for more than 1 year
  3. Voluntary participation in this research
(ii) Exclusion criteria
  1. Gui Peisheng
  2. Training nurse
  3. Those who cannot participate in the survey due to sick leave, personal leave, or going out for advanced studies or studies

### 3.2. Experimental Research Methods

The research process of this article mainly adopts the questionnaire survey method, including two questionnaires: one is a questionnaire about nurses' awareness of clinical alarms, and the other is a questionnaire for clinical alarm fatigue.

The influencing factors of nurses in the intensive care unit on medical equipment alarm fatigue mainly include the following factors: gender, marital status, education, position, title, working years, employment form, number of night shifts per month, and whether there is a habit of setting up medical equipment alarms.

Clinical Alarm Questionnaire: the questionnaire was originally formulated by the Healthcare Technology Foundation (HTF) in 2005, and a new clinical alarm investigation was conducted in 2011, and the questionnaire was revised based on the results. The Cronbach's *α* coefficient of the questionnaire used in this study was 0.83, and the validity was 0.86. The scale uses Likert 5-level scoring and assigns values based on scores.

The survey nurses' cognition of clinical alarms is based on the 19 items in the HTF survey in 2011. Each item is assigned a value of 1 to 5 points from “strongly disagree'” to “strongly agree.” The higher the score, the more the nurse agrees with the implementation of the project.

### 3.3. Data Collection

Consult the relevant departments of the hospital and contact the head nurses of the intensive care unit of four tertiary hospitals, explain to them the purpose and methods of this research, and ask the relevant departments of the hospital and the head nurses to issue questionnaires. The nurses who participated in the survey received the questionnaire, and the answering time can be adjusted according to their own rest time to ensure that the nurse under investigation has sufficient time to consider the questionnaire and ensure the quality of the questionnaire. 220 questionnaires were issued, 215 points were returned, and the recovery rate was 98%.

### 3.4. Statistical Methods

All data were compared and logically checked, and SPSS21.0 was used for statistical analysis after confirming that the data was entered correctly. The count data in the general data of nurses is described by frequency and percentage. The tested data are in accordance with the normal distribution, and the measurement data is described by the mean ± standard deviation; the comparison of alarm cognition and alarm fatigue scores uses *t*-test and one-way analysis of variance; multiple linear regression analysis was used to analyze the factors affecting nurses' alarm fatigue; *P* < 0.05 indicates that the difference is statistically significant.

## 4. The Current Situation and Influencing Factors of the Alarm Fatigue of Nurses' Medical Equipment in the Intensive Care Unit Based on Intelligent Medical Care

### 4.1. Awareness of Nurses' Medical Equipment Alarms

The results in Table 1 and Figure 2 show that, in the multifactor analysis of alarm cognition for nurses with different characteristics, different educational backgrounds have different cognition levels for alarm. Most of the nurses in the intensive care unit with college degree and no job are in the work of critically ill patients who directly contact the nursing staff, and provide bedside monitoring for the patients. They will be dealt with as soon as they find that the patient's condition changes. The design of clinical alarm should be prioritized according to the criticality of the alarm event, and the nurse judges the alarm by prompting. The alarm is distinguished from the sense of hearing and vision to make it unique and “directional,” which can remind the nurses more intuitively and clearly and ensure the safe and efficient conduct of clinical work.

From this survey, nurses all indicated that nuisance alarms interfere with patient care. Nurses with a large number of night shifts are physically stressed, and sleep time and sleep quality cannot be guaranteed, which can cause circadian clock disorders, endocrine disorders, neurasthenia, personal problems, etc. The nursing staff on duty at night is not adequately equipped, the workload is large, and it is easy to lose concentration, and the nuisance alarm has an important impact on the nursing work of nurses.

It can be seen from Table 2 and Figure 3 that items such as alarm sound, nuisance alarm interfering with patient care, inability to hear the alarm, and missed alarm are all statistically significant for the nurse alarm fatigue item.

Nurses with different characteristics have different cognitions of alarms. Among them, nurses with college degree and no job can recognize the importance of alarm sounds and visual prompts, and nurses with night shifts ≥11 days per month recognize that nuisance alarms interfere with nursing work. However, it is necessary to strengthen the training of low-age nurses' missed alarms, false alarms, and alarm management policies and new monitoring system awareness training. Nurses in the intensive care unit are suffering from severe alarm fatigue. We will strengthen the management and training of nurses who are married, have low academic qualifications, have low professional titles, have low working years, and have no habit of alarming, so as to improve their professional level and the quality of nursing services to provide protection for the safety of patients.

It can be seen from Table 3 and Figure 4 that, in the significance test of the path coefficient of perceived usefulness to use intention, the *P* value is less than 0.01, and the result is significant. Among the related assumptions about information quality, information quality has a significant impact on both perceived usefulness and perceived risk.

### 4.2. Influencing Factors of Alarm Fatigue of Nurses in the Intensive Care Unit

The lower the score, the greater the barrier to alarm management. Ranked first is the following: frequent false alarms make nurses less concerned about and respond to alarms, with a score of 3.55 points. The last in the ranking is lack of training on the alarm system, with a score of 6.40 points. See Table 4 and Figure 5 for details.

Alarm fatigue is a complex and uncontrollable cognitive process. It is the result of changes in human cognition and attention in order to adapt to the surrounding environment. Alarm fatigue cannot be simply regarded as an overcontact alarm. In the results of this survey, the total score of nurse alarm fatigue is 24.63 ± 8.99. It can be seen that the alarm fatigue of nurses in the intensive care unit is at a severe level, which needs to be taken seriously in the intensive care unit. The item with the highest score was “Clinical alarms made me stressful.” On the one hand, due to the large number of instruments and equipment in the intensive care unit and the large number of alarms, the nurse was overloaded when handling the alarm; on the other hand, it was the long-term exposure of the intensive care nurse The noisy alarm sound leads to auditory habituation, which in turn increases cognitive burden and psychological exhaustion. Nurses who have been in such a bad environment for a long time also increase their mental stress, and alarm fatigue is more likely to occur.

We take alarm fatigue score as the dependent variable, and marital status, educational background, position, title, working years, and the habit of setting medical equipment alarms as independent variables for assignment, as well as doing multiple linear regression analysis. It can be seen from Figure 6 and Table 5 that marital status, job title, working years, job title, the habit of setting up medical equipment alarms, and educational background are the main factors affecting alarm fatigue. Marital status has the greatest impact, followed by job titles. In addition, unmarried, high-level positions, long working years, high professional titles, and high education are negatively correlated with alarm fatigue (*P* < 0.05), and those without an alarm habit are positively correlated with alarm fatigue (*P* < 0.05), and the number of night shifts per month is related to the alarm.

The results in Table 6 and Figure 7 show that the orthogonal rotation is performed to obtain the factor loading matrix. The knowledge dimension includes basic knowledge of the alarm state of the ECG monitor (variance contribution rate 7.055%) and basic knowledge of the ventilator alarm state (variance contribution rate 4.852%); the belief dimension includes alarm positive belief (variance contribution rate 15.766%) and the cause of alarm fatigue (variance contribution rate 5.756%); behavior dimensions include alert parameters (variance contribution rate 4.601%), alert negative behaviors (variance contribution rate 9.647%), and alert positive behaviors (variance contribution rate 11.651%), roughly in line with the initial construction of the questionnaire. The questionnaire has good structural validity.

Grouped by the number of years of ICU nursing work, statistical analysis was performed on the three dimensions of ICU nurses' fatigue knowledge, beliefs, and behaviors of common monitor alarm response. The results are shown in Table 7 and Figure 8. The nurses with different nursing work years are obtained. The fatigue knowledge and behavior scores of commonly used monitors were statistically significant (*P* < 0.05). Nurses with different years of nursing work had no statistical significance in their commonly used monitors' alarm response fatigue belief scores (*P* > 0.05), pairwise comparison. The results showed that ICU nurses who worked for more than 11 years had higher fatigue knowledge and behavior scores in response to common monitor alarms than those who worked for 5–10 years and <5 years (*P* < 0.01); the trend test was taken as *α* = 0.05, knowledge dimension *F* = 15.319, *P*=0.001, belief dimension *F* = 2.287, *P*=0.104, behavior dimension *F* = 8.030, *P*=0.001.

According to the nursing profession satisfaction grouping, the ICU nurses' scores on the three dimensions of common monitor alarm response fatigue knowledge, belief, and behavior were statistically analyzed, and it was concluded that nurses with different nursing profession satisfaction, their common monitor alarm response fatigue beliefs, The behavior score is statistically significant (*P* < 0.05), and the common monitor alarm response fatigue knowledge score is not statistically significant (*P* > 0.05), as shown in the table; the pairwise comparison results show that the nursing occupation satisfaction is satisfactory for ICU nurses. The fatigue belief and behavior scores of common monitor alarm response are higher than those of nursing occupation satisfaction who are average and dissatisfied (*P* < 0.01); the trend test takes *α* = 0.05, knowledge dimension *F* = 18.661, *P*=0.001, belief dimension *F* = 7.611, *P*=0.001, behavioral dimension *F* = 9.873, *P*=0.001.

## 5. Conclusion

The main research in this paper is based on the analysis of the current situation and influencing factors of the alarm fatigue of nurse medical equipment in the intensive care unit based on intelligent medical care. Through the investigation and research on the nurses' alarm awareness and alarm fatigue in the intensive care unit of Y hospital, we further explore the current situation of intensive care unit alarm management, analyze its influencing factors, and provide a basis for perfecting the effective management of intensive care unit alarms and related nursing staff. The disadvantage of this article is that the investigation process is not strict enough, and the investigation data needs to be more perfected and supplemented. In the future, with the assistance of intelligent medical care, it can effectively improve the current situation of the alarm fatigue of nurses in the intensive care unit. According to its related influencing factors, we improve the accuracy of alarms, improve the quality of nursing services, and provide protection for the life safety of patients.

## Figures and Tables

**Figure 1:** Intensive care unit of a hospital.

**Figure 2:** Multifactor analysis of nurses' cognition of alarms with different characteristics.

**Figure 3:** Analysis of multifactor index of alarm cognition.

**Figure 4:** Perception scale and path coefficient analysis.

**Figure 5:** Score of alarm fatigue scale and alarm management disorder score of nurses in intensive care unit.

**Figure 6:** Multiple stepwise regression analysis of influencing factors of alarm fatigue of nurses in intensive care unit.

**Figure 7:** The characteristic value of each factor and the percentage explaining the total variation.

**Figure 8:** The influence of ICU working years and occupational satisfaction on the overall score of alarm response fatigue.

**Table 1:** Multifactor analysis of nurses' cognition of alarms with different characteristics.

Project		Alarm sound	Nuisance alarm	Missing the alarm	Clinical policies	Newer monitoring systems
*Gender*	Male	3.93	4.13	3.68	3.76	4.42
	Female	4.12	3.97	3.75	3.95	4.13

*Marital status*	Married	4.01	3.98	4.03	4.11	3.58
	Unmarried	4.03	4.12	3.99	3.92	4.09

*Education*	Junior college	4.23	3.74	3.98	4.02	3.69
	Undergraduate	4.11	4.12	4.45	3.94	3.26
	Master degree	3.72	4.11	3.97	3.85	3.33

*Job title*	Nurse	4.04	4.15	3.42	3.95	4.53
	Group leader	3.91	4.09	4.14	4.01	4.56
	Head nurse	3.45	3.95	3.76	3.58	4.28

*Working years*	1-2	4.00	4.05	3.15	4.08	3.59
	3–6	4.13	4.56	3.92	3.96	3.68
	7–11	3.96	3.78	4.01	3.75	3.79
	≥12	4.22	4.23	3.89	4.05	4.05

*Medical equipment alarms*	Yes	3.57	3.59	4.12	4.08	4.19
	No	4.12	4.28	4.13	3.85	4.23

**Table 2:** Analysis of multi-factor index of alarm cognition.

Project	*T* value	*P* value	*T*/*F* value	CR	AVE
Alarm sound	15.68	3.24	3.32	0.853	0.666
Nuisance alarm interferes with patient care	13.49	3.58	2.21	0.946	0.846
The condition of not hearing the alarm and missing the alarm	16.22	2.69	2.25	0.878	0.716
The institution has established effective clinical policies and regulations on alarm management	9.58	4.56	3.24	0.886	0.669
Newer monitoring systems can solve most of the old problems	12.24	4.55	3.33	0.895	0.764

**Table 3:** Perception scale and path coefficient analysis.

Scale information	Original sample	Sample mean	Standard deviation	*T* value	*P* value
Information quality	−0.451	−0.452	0.066	6.695	≤0.001
Perceived usefulness	0.415	0.418	0.087	4.692	≤0.001
Perceived risk	0.057	0.054	0.081	0.675	0.501
Willingness to use	−0.163	−0.163	0.632	2.596	0.010

**Table 4:** Score of alarm fatigue scale and alarm management disorder score of nurses in intensive care unit.

Entry	Score	Scoring rate (%)
The instrument alarm made me feel anxious A1	3.02	60.21
The instrument alarm makes it difficult for me to concentrate A2	2.98	59.62
The instrument alarm made me feel terrible A3	2.87	57.32
The instrument alarm makes it easy for me to forget what I had to do A4	2.66	53.62
The instrument alarm gives me a headache A5	2.53	50.41
The instrument alarm made me feel powerless A6	2.48	49.42
The instrument alarm makes me tired of everything A7	2.35	47.23
Total score A8	18.88	53.95
Frequent false alarms reduce nurses' attention and response to alarms B1	3.57	42.58
Difficult to understand the priority of alarms B2	3.98	51.36
It is difficult to hear the alarm when an alarm occurs B3	4.73	54.29
Insufficient number of staff responding to the alarm B4	4.78	57.83
Difficult to identify the source of the alarm B5	5.01	55.34
Difficulties in setting the alarm correctly B6	5.02	56.22
Overreliance on the alarm to draw attention to patient problems B7	5.41	59.87
Noise competition from nonclinical alarms and pages B8	5.98	53.91

**Table 5:** Multiple stepwise regression analysis of influencing factors of alarm fatigue of nurses in intensive care unit.

Variable	*B*	SE	*β*	*t*	*P*
Constant	6.533	2.936	—	19.257	<0.001
Marital status	−1.635	0.792	−0.881	−2.068	0.051
Job title	−8.384	0.758	−0.429	−10.782	<0.001
Working years	−3.435	0.524	−0.336	−6.654	<0.001
Job title	−3.233	0.587	−0.235	−5.158	<0.001
Do you have a habit of setting up medical equipment alarms?	4.865	0.936	0.191	5.256	<0.001
Education	−5.231	1.289	−0.158	−4.087	<0.001
Number of night shifts per month	<0.001	0.387	<0.001	<0.001	1.000

**Table 6:** The characteristic value of each factor and the percentage explaining the total variation.

Factor	Eigenvalues	The total variation	Accumulation
Positive attitude to the police, C1	3.943	15.766	15.766
Alarm positive behavior, C2	2.922	11.651	27.427
Alarm negative behavior, C3	2.419	9.647	37.055
Basic knowledge of ECG monitor alarm status, C4	1.765	7.055	44.118
Alarm fatigue reason, C5	1.448	5.756	49.862
Basic knowledge of ventilator alarm status, C6	1.223	4.852	54.724
Alarm parameters, C7	1.156	4.601	59.325

**Table 7:** The influence of ICU working years and occupational satisfaction on the overall score of alarm response fatigue.

Project		Knowledge standard score	Belief standard score	Behavior standard score	*F*	*P*
*ICU working years*	＜5	59.58	74.48	76.23	15.129	<0.001
	5–10	62.01	76.37	75.27	2.284	0.114
	＞11	85.15	79.74	85.23	8.031	<0.001

*Professional satisfaction*	Satisfaction	63.58	80.77	82.23	0.161	0.853
	General	62.73	74.41	75.72	7.622	0.001
	Dissatisfied	32.01	71.63	71.53	9.871	<0.001

## Data Availability

No data were used to support this study.
